The article "Analysis of Diabetes Clinical Data Based on Recurrent Neural Networks" was retracted in 2023. Reasons: signs of a paper mill; suspected computer-generated content; unreliable results or conclusions; lack of ethics approval or compliance.

# Analysis of Diabetes Clinical Data Based on Recurrent Neural Networks

**DOI:** 10.1155/2022/4755728

**Published:** 2022-06-27

**Authors:** Yuanyuan Lin, Yueli Li, Xuemei Huang, Li Liu, Haitao Wei, Xinyu Zou

**Affiliations:** Department of Endocrinology, First People's Hospital of Nanning, Nanning 530021, China

## Abstract

At present, diabetes is one of the most important chronic noncommunicable diseases, that have threatened human health. By 2020, the number of diabetic patients worldwide has reached 425 million. This amazing number has attracted the great attention of various countries. With the progress of computing technology, many mathematical models and intelligent algorithms have been applied in different fields of health care. 822 subjects were selected in this paper. They were divided into 389 diabetic patients and 423 nondiabetic patients. Each of the subjects included 41 indicators. Too many indicator variables would increase the computational effort and there could be a strong correlation and data redundancy between the data. Therefore, the sample features were first dimensionally reduced to generate seven new features in the new space, retaining up to 99.9% of the valid information from the original data. A diagnostic and classification model for diabetes clinical data based on recurrent neural networks were constructed, and particle swarm optimization (PSO) was introduced to optimise recurrent neural network's hyperparameters to achieve effective diagnosis and classification of diabetes.

## 1. Introduction

Diabetes is a common and highly prevalent disease that affects the entire body system in the world. According to the 2020 diabetes statistics, the number of diabetic patients in the world has reached 425 million. Recently, the number of diabetic patients worldwide continues to rise, and it is expected to reach 629 million [1] in 20 years. This means that in ten people, there are at least one people has diabetes. If diabetes is not diagnosed and treated in a timely manner, patients are also at increased risk of having diseases such as heart disease and diabetic nephropathy [2]. Huge amounts of money are spent globally on health care for diabetes each year, with total costs reaching $760 billion by 2019. This figure is expected to grow to $825 billion in 2030 and $845 billion in 2045 [3], with the largest global expenditure on the diagnosis and treatment of diabetes and its related diseases being in the USA, followed by China and Brazil. The 60–69 age group is the most affected by diabetes, followed by the 50–59 and 70–79 age groups, respectively. Diabetes also shows some gender differences, with a higher proportion of women with diabetes than men and is expected to continue along with current age trends and gender differences in the coming decades. The morbidity of diabetes is influenced by genetic factors and lifestyle habits and is highly likely to lead to macrovascular and microvascular complications leading to death and renal failures, such as cardiovascular disease and diabetic nephropathy, severely reducing the quality of life of patients [4, 5].

In the era of big data, mathematical models and algorithms are widely used to deal with real problems in various fields. Machine learning, neural networks, and intelligent algorithms have all become effective techniques for analysing clinical data on diabetes. Computer algorithms are widely used for the correct diagnosis and classification of diabetes. In the direction of machine learning, many scholars have established KNN models, LDA models, SVM models, decision trees, and random forests [6, 7] to classify and predict diabetes. In the direction of neural networks, Rabie et al. used neural networks to predict diabetes symptoms in a Chinese city [8]. Asghar et al. built three supervised learning prediction models to analyse and predict diabetes based on whether the patient has diabetes, including both machine learning methods and neural network methods, including support vector machines (SVM), k-nearest neighbours (k-NNs), and artificial neural networks (ANNs) [9].

The building of diagnostic models for diabetes can be summarised in three modules: first, feature selection based on preprocessed clinical data to obtain the most effective feature information; second, optimization of classification and prediction models in combination with intelligent optimization algorithms, with the optimized models usually achieving better classification and prediction results; third, analysis of diabetes clinical data using deep learning algorithms, including BP neural networks and DNN neural nets.

In this paper, 822 people were selected for clinical analysis, divided into diabetic and nondiabetic patients, and 41 test indicators of each study subject were used as feature variables. A recurrent neural network (RNN) based classification model for diabetes was developed by performing the principal component analysis (PCA) on the feature variables, combined with a particle swarm algorithm (PSO) to optimise the conventional RNN hyperparameters to achieve good diagnostic and classification results.

## 2. Methods

### 2.1. Principal Component Analysis (PCA)

When observing and analysing data, data sets in many fields contain numerous features. A larger amount of features can provide more detailed and comprehensive information, but it also increases the amount of computation and the difficulty of data analysis. When there are many data features, there is a high probability of correlation between variables, and if some of the features are randomly selected for analysis, the valid information in the data cannot be fully utilised, resulting in the loss and waste of valid information. PCA (principal component analysis) reduces data features and retains the original effective information of characteristic variables as much as possible [10], reducing information loss and eliminating correlations between features, in order to achieve a comprehensive analysis of the data.

The principle of PCA is to find a set of orthogonal axes in the original space in a sequential manner [11]. The first new axis is selected, which is based on the direction with the largest variance in the original data; the second new coordinate axis is selected in the plane orthogonal to the first coordinate axis to maximize the variance; the third axis has the largest variance in the plane orthogonal to the first two axes. The final n-dimensional features are mapped to the m-dimensional, and the newly generated m-dimensional features are referred to as the principal components. PCA is a preprocessing method [12]. It removes noise and some unimportant features, but the most important features will be retained. In this way, the speed of data processing will be greatly improved, and a lot of data analysis time and cost can be saved.

In diabetes clinical treatment and monitoring data, the same correlations exist between indicator variables, so consideration was given to eliminating correlations between different indicator characteristics, reducing the number of indicators so that the indicator variables are two-by-two uncorrelated, retaining valid information from the original diabetes clinical data, and using fewer composite indicators to represent each type of information in each diabetes clinical data indicator separately.  Figure 1 shows the mathematical principle of PCA as described in the web blog we borrowed.

The process of implementing PCA for diabetes clinical data is as follows. Assuming that the data set is represented as *X*, the dimensionality after weight reduction is *t*.

(1) $$\begin{array}{c} X=\left\{x_{1},x_{2},x_{3}\ldots x_{n}\right\}. \end{array}$$

Firstly, the characteristics of each index are centralized, that is, their average value is substracted; then, the covariance matrix 1/*nXX*^*T*^ is calculated, the eigenvalues and eigenvectors are calculated and the eigenvalues from largest to smallest are sorted. Retain the first *t* maximum features. Finally, the data is transformed into a new space *Y* consisting of *t* features.

(2) $$\begin{array}{c} Y=PX. \end{array}$$

### 2.2. Recurrent Neural Network (RNN)

In 1988, Ronald Williams and his colleague, David Zipser raised a new algorithm called real-time recursive learning of recurrent neural networks (RTRL). A year later, Paul Werbos came up with BP through time (BPTT) of recurrent neural network [13]. Both have been used to date as the main methods for RNNs.

Conventional neural networks consist of an input layer, an implicit layer, and an output layer, and although there are connections between the layers, the nodes within the layers are not connected [14]. As a result, many real-world problems cannot be handled using conventional neural networks. The advantage of RNNs is that the current output is associated with the previous output [15] and the network is able to memorise the output of the previous layer and apply it with the extremes and outputs of the current layer, which means that the hidden layers are connected to each other node-to-node. The input information of the current hidden layer is divided into two parts, including the output of the input layer and the output of the previously hidden layer. RNNs have more feedback input neurons than conventional neural networks, and their neurons resemble a series of sequential connections of weight-sharing feedforward neurons, with historical information from the previous moment connecting the next moment neurons in a weighted manner. Thus, the input of the RNN at moment *t* completes the mapping to the output and references all input data to the network before *t*, forming a feedback network structure, as revealed in Figure 2.

For a conventional feedforward neural network, the activation of node *t* at the moment is given by the following equation:

(3) $$\begin{array}{c} {\text{net}}_{j}\left(t\right)=\sum_{i}^{n}x_{i}\left(t\right)v_{ji}+\theta_{j}. \end{array}$$

Here, *n* means the number of nodes in the input layer and *θ*_*j*_ is the bias parameter. However, in RNNs, whether a node is activated or not is related to the input layer at the previous moment, as well as the hidden layer, the nodes of the hidden layer are “cyclically” used in the neural network. In this case, the activation formula for the nodes is updated as follows:

(4) $$\begin{array}{c} \left\{\begin{array}{c} {\text{net}}_{j}\left(t\right)=\sum_{i}^{n}x_{i}\left(t\right)v_{ji}+\sum_{i}^{n}h_{l}\left(t-1\right)u_{jl}+\theta_{j},\\ h_{l}\left(t\right)=f\left({\text{net}}_{j}\left(t\right)\right). \end{array}\right. \end{array}$$

Here, *m* refers to the total number of hidden layer nodes, at the same time, *f* is the activation function of the hidden layer nodes. Commonly used hidden node activation functions include sigmoid function and tanh function or binary function [16]. The output layer activation formula of RNN is

(5) $$\begin{array}{c} \left\{\begin{array}{c} {\text{net}}_{k}\left(t\right)=\sum_{j}^{m}h_{j}\left(t\right)w_{kj}+\theta_{k},\\ y_{k}\left(t\right)=g\left({\text{net}}_{k}\left(t\right)\right). \end{array}\right. \end{array}$$

Here, *g* is denoted as the activation function of the output layer node.

### 2.3. Particle Swarm Optimization (PSO) Algorithm

Particle swarm optimization (PSO) [17, 18] is an evolutionary computational technique that has been applied in a number of fields, stemming from the study of the behaviour of bird flocks foraging. PSO cooperates among individuals in the group and shares information to find the optimal solution [19]. The particle swarm optimization algorithm does not need to adjust many parameters, so it is easy to implement [20]. Therefore, it can be widely used in the application of genetic algorithms such as function optimization and neural network training. The particle swarm algorithm models each example as a massless bird in a flock of birds, including two attributes, velocity *v*_*i*_ and position *x*_*i*_.

(6) $$\begin{array}{c} \left\{\begin{array}{c} {\text{v}}_{i}=\omega \times {\text{v}}_{i}+c_{1}\times \text{rand}\left(\;\right)\times \left(p{\text{best}}_{i}-x_{i}\right)+c_{2}\times \text{rand}\left(\;\right)\times \left(g{\text{best}}_{i}-x_{i}\right),\\ x_{i}=x_{i}+{\text{v}}_{i}. \end{array}\right. \end{array}$$

Here, *ω* is a non-negative inertia factor, and the size of *ω* is related to the global and local search capabilities, the larger the *w*, the stronger the global search capability and the weaker the local search capability. rand() is a random number between (0,1); *c*_1_ and *c*_2_ are learning factors; the maximum value of *v*_*i*_ is *v*_max_, and if *v*_*i*_ is bigger than *v*_max_, then *v*_*i*_=*v*_max_.

## 3. Experiments

### 3.1. Data Preprocessing

The article firstly preprocessed the collected clinical data on diabetes, removing invalid samples, monitoring outliers, filling in missing values, etc., and finally retained the clinical data of 822 patients, each with 41 monitoring indicator variables, including age, height, weight, BMI, CHO, VAR00007, ALT, TG, HDLC, LDLC, SNP1, SNP2 SNP3, and SNP4. The sample consisted of 389 diabetic patients and 423 nondiabetic patients, and a diagnostic and analytical model of diabetes clinical data was constructed using 41 indicator variables as features, which is based on recurrent neural networks. The article uses the label “1” to represent diabetic patients and the label “0” to represent nondiabetic patients.

After preprocessing of the diabetes clinical data, Figure 3 shows the overall distribution of diabetic and nondiabetic patients regarding the characteristic variables CHO and BMI.

It can be seen from the figure that the BMI of most subjects is within the normal range, a few are thin or fat, and a few are obese, without severe obesity. Cho values are concentrated between 4 and 8. Between diabetic patients and nondiabetic patients, the distribution of BMI and CHO had no significant difference.

Height and weight are continuous characteristic variables. For these variables, the average filling method is used. Accordingly, the model filling method was used for age and the median filling method was used for LPA. As shown in Figure 4, the box diagram reflects the difference in the median, upper four, lower four, maximum and minimum of diabetes, and nondiabetic patients.

Discrete characteristic variables, such as features SNP1, snp2, SNP3, and snp4, are divided into three signal types: 1, 2, and 3. The mode filling method is adopted. The feature distribution after filling is shown in Figure 5.

### 3.2. Analysis of Diabetes Clinical Data Based on RNN

Based on the pretreatment experiment, this paper launches a diabetes based clinical data diagnostic analysis experiment based on a recurrent neural network. Since there are up to 41 characteristic variables in the original data, principal component analysis is carried out first; then, the reduced dimension data are introduced into the cyclic neural network training model, and the PSO algorithm can optimise model parameters. After dimensionality reduction, seven new principal components are generated in the new space, and the effective retention information of the original data reaches 99.9%; num_ layers, hidden_ size, num_ Layers, etc., are set. As the set of superparameters to be optimized in RNN model, combined with PSO algorithm, when *ω*=0.5, *c*1=*c*2=2, the model diagnosis effect is the best. From the experimental results, the effective resolution accuracy of the optimized model for diabetics was 0.875, and the classification effect was good. At the same time, PCA technology effectively improves the calculation speed, saves the calculation time, and accelerates the convergence speed of the model.

After PCA dimensionality reduction, when the generated new feature dimension is 7; that is, the original 41 features are transformed into 7 new variables, which can retain 99.9% of the original feature information, as shown in Figure 6.

After dimensionality reduction, the size of the interpretable variance carried by each new feature vector and the contribution rate of the information amount of each new feature vector to the interpretable variance of the total information amount of the original data are shown in Table 1. The first newly generated feature retains 97.93% of the effective information of the original data, and the interpretable variance reaches 43275.2341; that is, most of the information is effectively concentrated on the first feature.

Based on recurrent neural network's clinical data analysis of diabetes, experiments show that the PCA greatly increases the speed of the model and reduces the time spent on calculations. Using the original diabetes dataset to carry out the RNN based diagnostic experiment, time-consuming 271 ms, using the dimensionality reduction data training model and classification experiment, the running time is reduced to 212 ms, effectively saving 21.7% computing time. As shown in Figure 7.

The model classification results were compared with the measured diabetes clinical data to verify that the proposed method can effectively diagnose whether the study subjects have diabetes. Meanwhile, PSO has significantly improved the diagnostic accuracy of diabetes. After introducing the PSO algorithm to optimise the combination of RNN hyperparameters, the diagnostic accuracy of the clinical patients with diabetes was improved from 0.84 to 0.875, as shown in Figure 8.

In addition to Accuracy, we also used Precision, Recall values, and F1 values as measures of model performance, and Table 2 showed the results of each metric.

## 4. Conclusion

Diabetes is a metabolic disease of an infectious nature that directly affects the entire body system of the patient. Every year, hundreds of patients with diabetes suffer immensely. In the diagnosis and analysis of diabetes, the use of a historical patient information database to diagnose the disease based on the value of indicators of testing items has become one of the current effective technical means to detect and treat diabetes early to help maintain the healthy living of patients. These years, there has been a general trend to use machine learning and neural networks to build classification and prediction models for diabetes, and machine learning and neural networks can be used to distinguish whether the subject to be diagnosed is diabetic or not based on sample attributes. In the coming period, we will collect more clinical data on diabetes to validate and optimise the accuracy of the model, to better apply it to the diagnosis of diabetes patients with different characteristics such as gender, age, and region, and to compare the diagnostic results under different models.

## Figures and Tables

**Figure 1:** Mathematical principle of PCA.

**Figure 2:** RNN structure.

**Figure 3:** Distribution of the sample by gender.

**Figure 4:** Distribution of continuous features after filling.

**Figure 5:** Distribution of discrete features after filling.

**Figure 6:** Number of newly generated features of PCA.

**Figure 7:** Comparison of running time before and after PCA.

**Figure 8:** PSO optimization effect.

**Table 1:** Interpretable variance of new features after dimension reduction.

Features	Explained variance	Explained variance ratio
0	43275.2341	0.9793
1	713.5670	0.0161
2	81.8829	0.0019
3	57.3003	0.0013
4	19.9402	0.0005
5	14.9968	0.0003
6	8.5831	0.0002

**Table 2:** Evaluation indicators.

Accuracy	Precision	Recall	F1
0.875	0.875	0.89	0.88

## Data Availability

The data used to support the findings of this study are available from the corresponding author upon request.
